RETRACTED

# VSHR: A Mathematical Model for the Prediction of Second-Wave COVID-19 Epidemics in Malaysia

**DOI:** 10.1155/2022/4168619

**Published:** 2022-01-18

**Authors:** Xiang Yu, Lihua Lu, Jiangfan Guo, Haihuan Qin, Chunlei Ji

**Affiliations:** School of Electronics and Information, Shanghai Dianji University, Shanghai 201306, China

## Abstract

Since December 2019, a novel coronavirus (COVID-19) has spread all over the world, causing unpredictable economic losses and public fear. Although vaccines against this virus have been developed and administered for months, many countries still suffer from secondary COVID-19 infections, including the United Kingdom, France, and Malaysia. Observations of COVID-19 infections in the United Kingdom and France and their governance measures showed a certain number of similarities. A further investigation of these countries' COVID-19 transmission patterns suggested that when a turning point appeared, the values of their stringency indices per population density (PSI) were nearly proportional to their absolute infection rate (AIR). To justify our assumptions, we developed a mathematical model named VSHR to predict the COVID-19 turning point for Malaysia. VSHR was first trained on 30-day infection records prior to the United Kingdom, Germany, France, and Belgium's known turning points. It was then transferred to Malaysian COVID-19 data to predict this nation's turning point. Given the estimated AIR parameter values in 5 days, we were now able to locate the turning point's appearance on June 2^nd^, 2021. VSHR offered two improvements: (1) gathered countries into groups based on their SI patterns and (2) generated a model to identify the turning point for a target country within 5 days with 90% CI. Our research on COVID-19's turning point for a country is beneficial for governments and clinical systems against future COVID-19 infections.

## 1. Introduction

Since the day this new virus emerged, COVID-19 has attracted widespread research. Many scientists have attempted to explain its behavior from mathematical and dynamic modeling perspectives [1, 2], while others [3, 4] examined the relationship between government responses and the transmission speed of COVID-19. Reports from China [5] and Italy [6] have proven that effective government measures, such as school closings, travel restrictions, bans on public gatherings, emergency investments in health care facilities, contact tracing, and other interventions, are able to suppress or mitigate the spread of COVID-19. However, there existed no official indicator on these government measures before OxCGRT (the Oxford COVID-19 Government Response Tracker) [7] appeared. OxCGRT introduces 19 indicators into 3 categories: closure and containment, health, and economic support. It then keeps track of biweekly records of governmental measures and normalizes the score in the range [0,100]. To date, more than 2,000 research papers have referenced it as an official indicator of governmental measures.

RETRACTED

Although OxCGRT is frequently cited in COVID-19-related studies, it is seldom utilized in group behavior studies. The designers for OxCGRT indicate that many countries own similar OxCGRT patterns, probably because they took lessons from each other. This gave us an opportunity to observe the OxCGRT charts from countries with similar stringency index values, such as the United Kingdom, France, and Germany. Their similarities suggest that they adopt highly identical governmental measures and expect similar outcomes.

Some preliminary studies were carried out before mid-2020, and scientists were trying to find the relationship between government measures and the transmission parameters of COVID-19. In [8], Hale and his team attempted to decipher the mystery between the degree of government stringency and the death rate from COVID-19. In [9], Jayatilleke et al. carefully investigated the stringency index pattern of Sri Lanka and made a one-month prediction of future stringency indices. With this prediction, his team was able to forecast the incoming month's transmission trend of Sri Lanka. These studies, although innovative and inspiring, lacked data support at that time. The world was in the middle of the first COVID-19 infections, and governmental measures have not yet been validated for their results.

Another interesting yet unexplored topic for COVID-19 infection is how to predict the turning point in the future. A turning point is an important date when COVID-19 transmission enters an equilibrium state. This state is treated as a balance between the number of new infections and the number of recoveries, and it can be described mathematically as a point where the accumulated infections reach their maximum speed. In [10], researchers developed a mathematical model called RLIM to locate the turning point in New York, U.S.A., using a revised classical suspected infectious recovery (SIR) model and a 4^th^-order polynomial estimation to fit infection and recovery records. In [11], a segmented Poisson model was employed to predict COVID-19 outbreaks in Canada, France, Germany, Italy, the UK, and the US. In this article, the authors developed a novel COVID-19 transmission model named VSHR as a variant of the SIR model. This model takes vaccination records into consideration and defines an absolute infection rate *δ* to describe the transition probability between susceptible state *S* and total infection state *H*. In our model, *δ* plays a critical role, as it also serves as transferable knowledge and can be taught from a group of nations sharing similar SI patterns. Additionally, it is used for turning point prediction when its value drops into the range of other nations' turning points cluster.

RETRACTED

Since the absolute infection rate *δ* is the key in turning point estimation, a method with high precision is required to generate it from current data records. The autoregressive integrated moving average (ARIMA) model is chosen for our simulation data fitting method. In research work [12], scientists applied ARIMA to 145 countries to evaluate its performance. Simulation results from [12] indicated that the relative mean square errors (RMSE) from these countries were proportional to the population per million people. This conclusion strongly supports our assumption that ARIMA is able to provide stable and precise predictions of overpopulation density. The performance indicator in this article is the confidence interval (CI). In research work from [13], simulation results from Romania, Bulgaria, and Brazil prove that CI is an effective means in ARIMA's output evaluation. In VSHR, an evaluation of 90% CI is implemented to evaluate ARIMA's data fit quality.

In conclusion, VSHR is a model for COVID-19 transmission prediction. An absolute infection rate *δ* is calculated for a group of countries with similar SI patterns near their turning points' dates. This knowledge is then transferred to other nations' turning point predictions. To increase precision, a data fitting method called ARIMA is implemented, with a 90% CI. The main contributions of this approach are as follows:

1. Introduced a turning point indicator based on government control measure SI
2. Developed a mathematical model to locate the turning point of COVID-19
3. Validated the results with four countries: United Kingdom, France, Germany, and Belgium, successfully predicted the turning point for Malaysia with 90% CI

The rest of this article is organized as follows.  Section 2 discusses the necessary mathematical modeling, equations, algorithms implemented, and validation parameters.  Section 3 describes the simulation settings, software, and scientific packages utilized by the VSHR program. From Section 3.2, the authors analyze the COVID-19 data and simulation results for four European countries, and provides predictions on Malaysia's infections starting from mid-May, 2021.  Section 5 summarizes the work and brings further discussions.

## 2. Methods

In the first part of this section, we will introduce two key factors inside our model: PSI and AIR. After the presentation of these key notations, we propose our mathematical model named VSHR, which contains an infection epidemic dynamics model, and an ARIMA algorithm. In Section 2.3, a flow chart of VSHR is provided, and Algorithm 1 is given written in pseudocodes. We hope that readers obtain useful information on how data are processed and how a turning point's position is found.

RETRACTED

### 2.1. The VSHR Notations

We will introduce two notations that are essential in VSHR modeling and simulations: the personal stringency index (PSI) and the absolute infection rate (AIR).

#### 2.1.1. Personal Stringency Index (PSI)

The stringency index is calculated with the policy indicators C1–C8 and H1. The value of the index on any given day is the average of nine subindices pertaining to the individual policy indicators, each taking a value between 0 and 100:

(1) $$\begin{array}{c} \text{SI}=\frac{1}{9}\overset{9}{\underset{j=1}{\sum }}I_{j}. \end{array}$$

The personal stringency index (PSI) is defined as a dividend between the original value SI and the population density *M*:

(2) $$\begin{array}{c} \text{PSI}=\frac{\text{M}}{\text{SI}} \end{array}$$

In this paper, PSI is used as an indicator for turning point prediction. For readers who refer to this value in their research, please note that the value of PSI is only numerical and cannot be directly used as an indicator of government policy restriction evaluation, please refer to original SI records in your own research. In our model, PSI is proportional to the absolute infection rate (AIR) *δ*, as defined in Equation (3) (*δ* is defined in Equation (4)):

(3) $$\begin{array}{c} \frac{\text{PSI}}{\text{AIR}}=\text{constant}. \end{array}$$

#### 2.1.2. Absolute Infection Rate (AIR)

The absolute infection rate *δ* is calculated as the accumulated number of infections of the given day divided by the total susceptible group in the nation. It is a measurement of total infections in our model, VSHR, depicted by Equations (5) to (8). In the simulation, it is also an indicator of a nation's COVID-19 transmission trend, as shown in Figure 1. This parameter is calculated with a classical ARIMA method implemented in [12]. According to this value, we can predict the turning point of this target nation with a 90% CI.

### 2.2. VSHR: Mathematics

As is shown in Figure 2, VSHR is inspired by the classical susceptible infection recovery (SIR) model. First, we present the dynamics of our model with equations [4–7]:

(4) $$\begin{array}{c} \frac{{dS}_{t}}{dt}=-\delta_{t}\times S_{t}, \end{array}$$

(5) $$\begin{array}{c} \frac{{dH}_{t}}{dt}=\left(\delta_{t}\times S_{t}-\gamma \right)\times H_{t}, \end{array}$$

(6) $$\begin{array}{c} \frac{d{\text{V}}_{t}}{dt}=\rho \times S_{t}, \end{array}$$

(7) $$\begin{array}{c} \frac{{dR}_{t}}{dt}=\gamma \times H_{t}. \end{array}$$

Compared with the traditional model, VSHR has made the following modifications:

Add a status *V* to represent the vaccinated group: citizens in this group are considered immune against COVID-19 infections, so they are removed from the susceptible group (S).

RETRACTED

Modify status *I* into *H* to represent the accumulated infection cluster: people in Group *H* are considered the total population identified since the first day of COVID-19 infections within this nation.

Use parameter *δ* as a transition parameter between status *S* and *H*. As a critical factor within VSHR, the absolute infection rate is responsible for two important tasks: indicate the turning point for a target nation together with SI and serve as an optimization objective within the algorithm. Readers may consider it a starting point of VSHR as well as a termination criterion.

In algorithm implementation, the following assumptions are made:

The number of susceptible Group *S* on a given day follows Equation (8):

(8) $$\begin{array}{c} S_{t}=M-H_{t-1}-V_{t-1}. \end{array}$$

The number of vaccinated Group *V* on a given day is given by Equation (9):

(9) $$\begin{array}{c} V_{t}=V_{t-1}+k. \end{array}$$

In Equation (8), the number of susceptible groups is calculated as the total population of a target country minus yesterday's total accumulated infections and total vaccinated citizens. The number of total vaccinations was calculated by Equation (10). Readers may take care, as Equation (9) is only effective in predictions when real vaccine injection records do not exist. Additionally, interpolation was applied when vaccination records were missing or lost. In the simulation, we adopted linear interpolation to fill in missing values of these nations' vaccination records. For example, in the fourth column in Table 1, the values for *V*_*t*_ from May 26 to June 6 are also generated by the linear interpolation technique using Equation (10). Although vaccination records may not vary in linear formation, we assume that within 10 days, its behavior is approximately linear.

### 2.3. ARIMA Model

An ARIMA model assumes that its input is a series of time-dependent data points, and through its execution, the model is able to reveal the statistical and reliable meaning of these values. In our simulation, ARIMA requires three inputs: infection records *H*_*t*_, vaccination records *V*_*t*_, and starting date *T*_0_ (readers may refer to Table 2). Then, an ARIMA model is initiated with three parameters (*p*, *d*, *q*), where *p* is the order of autoregression, *d* is the degree of difference, and *q* is the order of the moving average [10]. In our simulation, the fitted data series in *H*_*t*_ is expressed in

(10) $$\begin{array}{c} H_{t}=\alpha +\overset{T_{0}}{\underset{i=1}{\sum }}\Phi_{i}\times H_{t-i}-q. \end{array}$$

The predicted data series in *H*_*t*,*p*_ is described in

(11) $$\begin{array}{c} H_{t,p}=\alpha +\overset{T_{0}+5}{\underset{i=T_{0}}{\sum }}\Phi_{i}\times H_{t-i}-q. \end{array}$$

RETRACTED

### 2.4. VSHR: Algorithm

Given the notations of the PSI, AIR, and ARIMA methods introduced, Section 2.3 summarizes the VSHR algorithm's execution process in Figure 3 to provide an overview of this model. Then, a pseudocode is provided for readers who have intentions to reproduce our experiments.

#### 2.4.1. VSHR Algorithm

The flow chart of the VSHR model is shown in Figure 1. The inputs for VSHR are as follows: (1) starting date and (2) country name. The databases utilized in VSHR are (1) SI database and (2) COVID-19 infection and vaccination database. These data records are publicly available in our GitHub repository [14]. Then, VSHR calls two subprocesses: PSI calculation and AIR calculation. Both subprocesses return specific PSI value series and AIR value series of the target country starting from the current date. The returned outputs are then compared with historical PSI and AIR values of the target group (UK, France, Germany, and Belgium). If the PSI and AIR values of the target country are within the range of this group, VSHR will initiate turning point estimation. The ARIMA method requests the previous thirty days of infection and vaccination records from the database as a training set and will provide ten-day predictive values with 90% CIs. With these predictive data records, VSHR is able to locate the turning point's position.

#### 2.4.2. Algorithm: VSHR

The pseudocode to calculate the turning point in VSHR is shown in Algorithm 1.

## 3. Experimental Settings

In this section, the authors present our simulations in the following order: in Section 3.1, we introduce the GitHub repository, which contains datasets and codes for implementation. In Section 3.2, we introduce necessary scientific packages and languages utilized in VSHR.

### 3.1. Data Source

The original data sources in our simulation are from [15, 16]. The dataset used in our simulations is stored in five CSV files, each containing one month of accumulated infection data and ten days of prediction data for our target countries. The data records are also shown in Tables 3 and 4. These CSV files are all stored in our GitHub repository [14]. Our software is publicly available on GitHub as well, with all codes and implementations available for research.

RETRACTED

### 3.2. Software Implementation

The programming language inside VSHR is PYTHON version 3.7, and the essential software package used is SCIPY version 1.5.4. Two software modules are inherited from SCIPY: integrate and optimize. VSHR utilizes the integrate function to calculate the MSE and optimize the function to fit the real infection data into a time series.

## 4. Simulation Results

In this section, simulation results are demonstrated in two parts.  Section 4.1 first introduces VSHR simulation outputs on four regions whose turning points are already known. Readers may refer to Figure 1 and Table 3 to obtain information on VSHR-simulated values, AIR, and accumulated infections. Then, we publish our predictive values for Malaysia in Figure 4 and Table 4, whose turning point is not yet known.  Section 4.2 explains how VSHR locates the turning point of Malaysia based on knowledge from other nations within the same group. The process of how turning points are clustered, when we initiate the predictions and finally lock down Malaysia's turning point, is fully explored.

### 4.1. Data Fit for the UK, France, Belgium, and Germany

The simulation outputs in VSHR for the United Kingdom, France, Germany, and Belgium are shown in Figure 1. VSHR will read in datasets from these nations according to the initial configurations given in Table 2. After datasets are loaded, the algorithm divides them into training sets and test sets and sets random values for the ARIMA method. ARIMA then sets up a model and calculates the fitted values on train set records. Then, it returns the AIR series for VHSR with a 90% confidence interval.

Considering that the ARIMA method does not have the ability to recognize the turning point, a knowledge transfer on VSHR is necessary. For example, on January 8^th^, United Kingdom's COVID-19 infections had reached their maximum increasing speed. In VSHR, the actual accumulated infections, *H*_*t*_, are labeled in the dataset, and the AIR of this date, 0.0463, will be stored for Malaysia's predictions. This specific value of AIR came from ARIMA's data fitting outputs before and after five days of this turning point's date (in the case of the United Kingdom, January 4^th^ to January 12^th^) (Tables 1 and 2).

Table 3 provides a better view of data simulation outputs from VSHR because it contains five elements: date, *H*_*t*_, *H*_*t*,*p*_, *V*_*t*_, and AIR. VSHR loads accumulative infection records into variable *H*_*t*_, and then, it loads accumulative vaccination records into variable *V*_*t*_. It then establishes a model with the preset configuration (*p*, *d*, *q*) and optimizes the variance between its outputs *H*_*t*,*p*_ and the real data records in *H*_*t*_. When optimization reaches a satisfactory point, VSHR stops execution and prints the final outputs. Based on the output *H*_*t*,*p*_ and the vaccination record in *V*_*t*_, the *AIR* can be calculated using Equation (5).

RETRACTED

In Table 4, simulation reports on the accumulated number of infections for Malaysia from May 16^th^ to June 6^th^ are given. Similar to Table 3, the output values included *H*_*t*_, *H*_*t*,*p*_, *V*_*t*_, and AIR. In addition, *V*_*t*,*p*_ was provided from May 27^th^ to June 6^th^ as vaccination predictions. Additionally, the values of *H*_*t*,*p*_ and AIR during this period were in the form of a range, from the lower limitation to the upper limitation. This is because of the confidence interval set as ninety percent. The simulations were complete before May 27^th^, so readers may verify the difference based on future Malaysian COVID-19 infection reports.

### 4.2. The Turning Point

To determine the turning point of Malaysia, the study of national AIR/PSI patterns is needed. VSHR needs to read in the global dataset of COVID-19 infections in GitHub [14], extract accumulated infections and accumulated vaccine columns from this dataset, and calculate the AIR values of the target nations. Our simulation was performed prior to Malaysia's turning point's occurrence, so we have no information on this date. However, VSHR also calculated the AIR values and PSI values for nations belonging to the same group of Malaysia: the UK, France, Germany, and Belgium. After VSHR performed data analysis on these countries, it returned a series of AIR/PSI values. Compared with our knowledge on turning points' dates for these nations, VSHR is now able to justify a region where a turning point is most likely to occur. The simulation results are displayed on Figure 4.

With the values in Table 3 being settled down, we are now able to determine the relationship between PSI and AIR in this group, as shown in Figure 4. Additionally, readers may refer to the third and fourth columns of Table 2 as well as the fifth column in Table 3 to determine their relationships. The AIR for the United Kingdom is in the range of 0.046 ± 0.004, and the PSI of the United Kingdom within January 4^th^ to January 12^th^ is a constant value of 3.4283; thus, within 10 days, the AIR/PSI value for the United Kingdom is 0.0134 ± 0.0011. The same calculation step produces the AIR/PSI value for Germany as 0.0137 ± 0.0001. Thus, we can decide that when a country's AIR/PSI value approaches 0.0135 and continues to increase; its turning point may appear within 5 days.

A further discussion is presented here regarding the speed and steepness of the turning point's occurrence. From Figure 4, readers may observe that the United Kingdom and France's AIR/PSI curves are quite smooth and regular. For Belgium and Germany, the shapes of their curves are quite irregular and steep. We suspect that the shapes of AIR/PSI curves are affected by geographic factors and seasonal parameters. The United Kingdom and France entered an equilibrium state in Winter, when Christmas was approaching. This reduced residents' outside activities as well. In the case of Germany and Belgium, their turning points appeared around April 2021, so government measures may be less effective against citizens' activities.

RETRACTED

## 5. Conclusion and Future Work

This research proposes a method to predict a country's turning point in COVID-19 infections. This method learns from a group of nations whose turning points are already known, shares similar stringency index patterns, and transfers knowledge to a specific country whose COVID-19 infection has not yet hit a turning point. Based on assumptions that nations within the same group have similar PSI/AIR values on dates near their turning points, a model named VSHR is implemented to assist turning point prediction. In the simulation, VSHR learned from the United Kingdom, Germany, France, and Belgium and successfully estimated the turning point date of Malaysia on June 2^nd^, 2021.

Currently, VSHR's capability of turning point estimation is limited because its database only contains information from five countries. Once a complete scanning of all 145 regions' information is complete, VSHR should be able to predict multiple scenarios.

The other field of application is to explore the relationship between PSI and ARIMA parameters (*p*, *d*, *q*). Currently, the calculation of PSI values and ARIMA simulations are independent. If PSI can be simulated as a time series by ARIMA, the precision level may increase as well.

## Figures and Tables

**Figure 1:** VSHR simulation outputs: UK (a), France (b), Belgium (c), and Germany (d).

**Figure 2:** VSHR model diagram.

**Figure 3:** VSHR diagram.

**Figure 4:** (a) AIR/PSI values for countries belonging to Group A. (b) AIR/PSI values for Malaysia's turning point (estimation).

**Algorithm 1:** VSHR algorithm.

**Table 1:** ARIMA model results (the UK to Malaysia).

Country	ARIMA		
	*p*	*d*	*q*
United Kingdom	7	0	0
Germany	4	0	0
France	2	0	0
Belgium	7	0	1
Malaysia	3	1	0

**Table 2:** VSHR simulation reports (the UK to Malaysia).

Country	TP date	SI	Population density
United Kingdom	2021/1/8	79.6	272.898
Germany	2021/4/28	75	237.016
France	2020/11/2	78.7	122.578
Belgium	2021/3/27	62.96	375.564
Malaysia	2021/5/31	80.56	96.254

**(a):** 

UK					Belgium				
Date	*H*_*t*_	*V*_*t*_	*H*_*t*,*p*_	AIR	Date	*H*_*t*_	*V*_*t*_	*H*_*t*,*p*_	AIR
01/04	2721626	0	2704116	0.042895	03/23	842775	1582996	912256	0.079594
01/05	2782713	0	2771295	0.043751	03/24	849090	1644497	918407	0.080285
01/06	2845269	0	2830587	0.044604	03/25	854608	1721719	929025	0.080908
01/07	2898056	0	2897009	0.045452	03/26	860731	1790211	932523	0.081588
01/08	2966248	0	2966451	0.046291	03/27	866063	1812308	944653	0.082152
01/09	3026346	0	3035938	0.047120	03/28	870757	1814642	947405	0.082636
01/10	3081372	2677971	3085348	0.047937	03/29	872936	1838047	952528	0.082879
01/11	3127647	2843815	3171173	0.048740	03/30	876842	1869875	954299	0.083306
01/12	3173295	3067541	3234968	0.049526	03/31	882453	1954192	960331	0.083951

**(b):** 

France					Germany				
Date	*H*_*t*_	*V*_*t*_	*H*_*t*,*p*_	AIR	Date	*H*_*t*_	*V*_*t*_	*H*_*t*,*p*_	AIR
10/29	1329820	0	1356519	0.020077	04/24	3291293	25319032	3192840	0.042217
10/30	1379294	0	1408038	0.020840	04/25	3306692	25602047	3218392	0.042438
10/31	1414364	0	1444605	0.021381	04/26	3312653	26029056	3270519	0.042542
11/01	1460543	0	1492813	0.022095	04/27	3338564	26811998	3310499	0.042932
11/02	1566634	0	1603822	0.023738	04/28	3366827	27929958	3334797	0.043374
11/03	1639235	0	1679994	0.024865	04/29	3391039	28867269	3362130	0.043752
11/04	1593159	0	1631631	0.024149	04/30	3405365	29663973	3381502	0.043990
11/05	1650965	0	1692315	0.025048	05/01	3423900	29997085	3364653	0.044260
11/06	1711917	0	1756417	0.025996	05/02	3432676	30259137	3390112	0.044393

RETRACTED

**Table 4:** VSHR simulation report on infections, Malaysia, May 2021.

Date	*H*_*t*_	*V*_*t*_	*H*_*t*,*p*_	AIR	Date	*H*_*t*,*p*_ (90% CI)	*V*_*t*,*p*_	AIR (90% CI)
05/16	470110	1915824	469954	0.0148	05/27	(543628, 545070)	2765624	(0.01737, 0.01742)
05/17	474556	1976085	474364	0.0149	05/28	(550536, 553404)	2820531	(0.01759, 0.01769)
05/18	479421	2052636	478964	0.0151	05/29	(557362, 561813)	2875439	(0.01782, 0.01796)
05/19	485496	2303580	485259	0.0153	05/30	(564041, 570307)	2930346	(0.01803, 0.01823)
05/20	492302	2384183	492122	0.0155	05/31	(570591, 578865)	2985254	(0.01825, 0.01851)
05/21	498795	2444780	498627	0.0157	06/01	(577031, 587478)	3040161	(0.01845, 0.01879)
05/22	505115	2489988	504925	0.0159	06/02	(583367, 596140)	3095069	(0.01866, 0.01907)
05/23	512091	2535975	511843	0.0162	06/03	(589602, 604844)	3149976	(0.01886, 0.01935)
05/24	518600	2630984	518322	0.0164	06/04	(595743, 613585)	3204884	(0.01906, 0.01963)
05/25	525889	2730536	525777	0.0166	06/05	(601794, 622364)	3259791	(0.01926, 0.01992)
05/26	533367	2730536	533222	0.0169	06/06	(607760, 631171)	3314699	(0.01945, 0.02020)

## Data Availability

The data used to support the findings of this study have been deposited in the GitHub repository (https://github.com/GJF-outlier/COVID_19).
